# Tackling Explicit Material from Online Video Conferencing Software for Education Using Deep Attention Neural Architectures

This article has been retracted.

**DOI:** 10.1155/2022/6334802

**Published:** 2022-05-11

**Authors:** Yongzhao Yang, Shasha Xu

**Affiliations:** Zhengzhou Preschool Education College, Zhengzhou, Henan 450000, China

## Abstract

The spread of the COVID-19 pandemic affected all areas of social life, especially education. Globally, many states have closed schools temporarily or imposed local curfews. According to UNESCO estimations, approximately 1.5 billion students have been affected by the closure of schools and the mandatory implementation of distance learning. Although rigorous policies are in place to ban harmful and dangerous content aimed at children, there are many cases where minors, mainly students, have been exposed relatively or unfairly to inappropriate, especially sexual content, during distance learning. Ensuring minors' emotional and mental health is a priority for any education system. This paper presents a severe attention neural architecture to tackle explicit material from online education video conference applications to deal with similar incidents. This is an advanced technique that, for the first time in the literature, proposes an intelligent mechanism that, although it uses attention mechanisms, does not have a square complexity of memory and time in terms of the size of the input. Specifically, we propose the implementation of a Generative Adversarial Network (GAN) with the help of a local, sparse attention mechanism, which can accurately detect obscene and mainly sexual content in streaming online video conferencing software for education.

## 1. Introduction

Going through the second wave of the digital age, humanity is now called upon to manage the multilevel social effects that arise through the ever-accelerating growth of the Internet. At the international level, efforts are being made to establish an institutional framework for protecting minors using new technologies. But as children's use of the Internet and new technologies are constantly evolving, few countries have implemented a fully operational framework in enacting regulations for illegal behaviors exclusively in the Internet environment. The harmonization of the laws of the nations is an essential precondition for the effective transnational treatment of cybercrime and the protection of minors. The prevention and response initiatives proposed as good practices by experts and stakeholders focus on children, parents, and educators, whose effectiveness is constantly being explored because Internet issues are continually evolving [1–3].

Obscene and mainly sexual content, such as pornography, is not allowed in applications accessible to minors, primarily in educational environments. In general, the modern legal framework imposes strict policies on nudity and sexual content, especially when it relates to children. Implementing these policies from a technological point of view is mainly based on the development and implementation of techniques (filters) that implement these policies. Corresponding techniques are applied internationally in the educational networks of many advanced countries and prevent with significant success rate access to sites belonging to categories such as: “porn” (sites with pornographic content), “gambling” (gambling sites), “drugs” (websites promoting drugs), “aggressive” (websites promoting aggressive behavior and racism), and “violence” (websites promoting violence) [4]. Because websites are categorized in the above categories using an automated process (due to the vast number of websites on the Internet), a website can be ranked incorrectly. For this reason, every educational organization follows international practice. It enables its users to inform the competent technicians when they find any malfunction of the service, who now manually correct the database that should be excluded.

In addition, social media giants enforce strict policies and established procedures for dealing with content and any harmful behavior, prohibiting content that endangers minors [5]. These include sexual harassment, abuse, and harmful and dangerous acts, uploading, streaming, commenting, engaging in activities that harm children, etc. Also, in recent years, these companies have become significant investors in the design of systems that detect sexually explicit material on the video clearly and effectively to prevent the release of material with unacceptable content [6].

The huge unresolved issue now is in cases of intentional or unintentional exposure to sexual content when using real-time video conferencing software, such as online video conferencing software, used extensively during the pandemic. In these cases, where content and streaming occur in real-time, it is challenging to detect obscene or sexual content, so there is no protection for underage students [7].

Obscene and primarily sexual content can be detected in streaming online video conferencing software for education with great precision. Based on the gap presented in the procedures and minors' risks, mainly students, this paper proposes an innovative deep attention neural architecture system to tackle explicit material from online education video conference applications. It is an advanced machine learning technique, precisely computer vision, which uses an intelligent attention mechanism that does not have a square of memory and time complexity in terms of the size of its input data. Specifically, the implementation uses a GAN, with the help of a local, sparse attention mechanism, of complexity O($n\sqrt{n}$). We take advantage of the probability distributions generated within this particular attention mechanism while maintaining the 2d geometry of the multimedia content.

## 2. Related Literature

The literature concerning the field of detection mechanisms concerning specific or explicit content [1, 3] is varying due to the different approaches that the research community has:

Li et al. [8] studied numerous motion classification algorithms, concentrating on video using classifiers, mostly frame-based. They divided the basic processes into three main categories: the first was frame-by-frame recognition, the second was extracting sequences, and the third was temporal-information monitoring, which used the LSTM structure or the optical flow approach to remove training data between sequences. They also divided and characterized the various types of deep learning-based cameras as follows: Convolutional Neural Networks-based methods, Restricted Boltzmann Machine-based methods [9], and Autoencoder-based techniques, all examples of unsupervised ML algorithms that could acquire the representations and produce data frames with similar attributes.

Longlong et al. [10] looked at self-supervised generic image learning techniques based on deep learning from media files. They defined the key terms and examined the most prevalent self-supervised learning deep neural network topologies. They next looked at the architecture and evaluation criteria for self-supervised learning techniques, as well as the most often used samples, primarily for videos, and current self-supervised visual feature learning techniques [11]. They examined the practices of the shapes on image and video feature learning benchmark datasets. They finished their proposal by outlining several potential avenues of development for self-supervised visual feature learning.

Arachchi et al. [12] introduced a state-exchanging long short-term memory (SE-LSTM) two-stream neural network approach, based on the benefits of using spatial and motion information to identify dynamic patterns. This method was used to identify movie reactions using appearance motion characteristics. It could also be used to expand the general purpose of LSTM by sharing data with past cell states in both the look and action streams. The movies could not include any other active items than the target objects to achieve better classification performance, and the contexts had to be static [13]. The trial findings showed that the technique surpassed other collections in precision, particularly when it came to static background dynamic patterns classifications. To decrease discrepancies, they proposed eliminating all mislabeled information in the next round of their study.

Duboyskii et al. [14] used automated emotional state recognition and video conferencing technologies to transmit distant material in travel communication systems, surveys, and other applications. They created a peer-to-peer framework for remote communication sessions, allowing clients to share audio and visual information. At the operator end, convolutional neural networks were used for stream processing and to evaluate the customer's emotional responses. Three mechanisms (video, audio, and text) and multimodal recognition were employed to establish the dynamic conditions. The test was carried out between persons in which one served as an operator and posed closed questions while the other answered them. The proposed technology could be used in various sectors, including service delivery and healthcare, where real-time human emotion identification is essential. The neural network produced the highest accuracy values when multimodal recognition was applied, indicating its effectiveness in video conferencing systems for classifying human emotions. Their system had the disadvantage of only supporting one-to-one user connections, which they plan to address by expanding the number of concurrent user connections.

In 2016, Vondrick et al. [15] introduced a generative adversarial network for films using a Spatio-temporal convolutional architecture that untangled the scene's images by investigating how to learn behaviors from vast volumes of unstructured camera footage. It is expected that the scene dynamics will be critical for the next phase of computer vision systems and learning from unlabeled data would be a promising option. Tests and simulations revealed that the model recognized important aspects for detecting actions with little control on the inside. Despite the fact that fully realizing the potential of unlabeled video is still a work in progress, their findings suggest that having a lot of unsupervised videos might be beneficial for both training to create films and acquire graphical images.

Tulyakov et al. [16] proposed the Motion and Content deconstructed Generative Adversarial Network (MoCoGAN) framework for motion and content decomposed video production using the Generative Adversarial Network. In an unsupervised fashion, the MoCoGAN was trained to distinguish signal from content, and a movie was created by mapping a set of random vectors to a set of image sequences. They presented a unique adversarial learning method that learned motion and content decomposition unsupervised using both image and video discriminators. A Gaussian distribution was used to describe the content subspace, while a recurrent neural network to model the motion domain. The efficiency of the suggested framework was confirmed by experimental findings on datasets with qualitative and quantitative comparisons to state-of-the-art techniques [17]. They also demonstrated how their scheme could be used to produce videos with the same material but distinct motion, as well as films.

To overcome the short sample issue in hyperspectral image classification, Feng et al. [18] presented a symmetric convolutional GAN based on collaborative learning and attention mechanism (CA-GAN). A combined spatial-spectral intricate attention module was used in the Generator to filter out misleading and confusing aspects of the produced samples and force the distribution of generated models to resemble the pattern of genuine hyperspectral images. To retrieve combined spatial-spectral information of images, a convolutional LSTM layer was fused in the Discriminator. In addition, by using the actual sample information retrieved by the Discriminator, a collaborative learning process was devised to aid sample production in the generator. It allowed the Generator and Discriminator to be refined alternately and collaboratively via competition. Tests on noteworthy sources of data revealed that their method outperformed the other approaches in terms of classification accuracy, particularly when the number of training samples was restricted. The studies indicated that they will look into more efficiently and automatically determining the placements and numbers of different modules, and they will experiment with different sampling methods to eliminate overlap between training and testing sets.

From the literature mentioned, we see that the research community is actively focusing on finding methods and techniques to increase the performance of media classification, according to the specific needs of each individual Case [3, 19].

## 3. Methodology

The proposed implementation is based on the GANs architecture [18, 20], which uses an optimal local, sparse attention mechanism. Using a previous frame's context, a video prediction algorithm can foretell the next frame in a video. Unlike a static image, a video allows the viewer to see the changes and motion patterns over a more extended period. For this reason, the model must take into account both time and space to accurately predict the future frames in a video. Modeling temporal dynamics is typically done using Recurrent Neural Networks. However, GANs have become the most popular method for predicting future video frames. A vital element of the structure of GANs is the existence and simultaneous training of two networks, the Generator that creates samples as close as possible to those of the training set and the Discriminator that is trained to distinguish which samples come from the training set (i.e., are they real) and which one from the Generator (i.e., are they artificial or fake). Specifically, at each training Step (i.e., inside the training loop), the Discriminator receives samples from the training data set and samples generated by the Generator and is trained to have a probability of close to 1 for the first and close to 0 for the second. In contrast, the Generator is trained so that from input noise to output images to the output realistic enough to “trick” the Discriminator.

Going a little deeper into the analysis of how GANs are trained, we can say that both Generator and Discriminator are represented by (continuously) differentiable functions with trainable parameters, such as neural networks, each with its cost function. The two networks are trained through back-propagation using the Discriminator cost function, but with a different goal. The Discriminator tries to reduce the cost function for both natural and artificial samples, while Generator tries to increase the Discriminator cost function for the synthetic samples it produces. It is noteworthy that the training data set alone determines the type of samples that the Generator learns to create.

The Binary Cross-Entropy cost function is used in the proposed methodology. For each predicted probability, Binary Cross Entropy compares it to the class output of 0 or 1. Once the score has been calculated, probabilities are penalized based on the distance from the expected value. This is a measure of how close or how far the calculated value is from the actual value. Specifically, for a set of *m* samples per batch is as follows [17]:

(1) $$\begin{array}{c} J_{m}23\left(\overset{⟶}{\partial }\right)=-\frac{1}{m}\overset{m}{\underset{i=1}{\sum }}\left[y^{\left(i\right)}\log\left(h\left(x^{\left(i\right)};\overset{⟶}{\partial }\right)\right)+\left(1-y^{\left(i\right)}\right)\log\left(1-h\left(x^{\left(i\right)};\overset{⟶}{\partial }\right)\right)\right], \end{array}$$

where the initial sum and division by the number of samples approximates the mean value operator, *x*(*i*) is the *i*-th sample, *y*(*i*) is the label of the *i*-th sample, and ∼*θ* is the vector of the trainable model parameters. During the Discriminator training of the proposed GAN, the labels will be 1 for the actual samples and 0 for the artificial ones. In contrast, for the training of the Generator, the reverse is true, i.e., together with the synthetic samples, label 1 will be given to calculate whether it may “trick” the Discriminator.

Focusing on the formation of the cost function and the values it receives for the 0/1 tags given during the training of a GAN, we see that when the tag is 1, only the first term of the sum acts. Considering the negative sign at the beginning of the equation, we see that the above Binary Cross-Entropy approach for a batch takes values from 0 to +∞ when the classification function *h*(*x*) with parameters *θ* takes values from 0 to 1.

Optionally, the Binary Cross Entropy cost function has two parts (one for each class) and takes values close to 0 for correct configuration (diagonal confusion matrix) while approaching the positive infinity for error (diagonal confusion matrix) - behavior graphically illustrated in Figure 1 below [17]:

Thus, for the Discriminator, the Binary Cross-Entropy cost function given that during GAN training, the actual data is contractually assigned the tag 1 and the artificial data to 0, will be [17]:

(2) $$\begin{array}{c} \begin{array}{c} J_{D}\left(\overset{⟶}{\partial_{D}},\overset{⟶}{\partial_{G}}\right)=-\frac{1}{m}\overset{m}{\underset{i=1}{\sum }}\left[y^{\left(i\right)}\log\left(h\left(x^{\left(i\right)};\overset{⟶}{\partial }\right)\right)+\left(1-y^{\left(i\right)}\right)\log\left(1-h\left(x^{\left(i\right)};\overset{⟶}{\partial }\right)\right)\right]\\ =-\frac{1}{m}\overset{m}{\underset{i=1}{\sum }}\left[\log\left(D\left(x^{\left(i\right)};\overset{⟶}{\partial_{D}}\right)\right)+\log\left(1-D\left(G\left({\overset{⟶}{z}}^{\left(i\right)};\overset{⟶}{\partial_{G}}\right);\overset{⟶}{\partial_{D}}\right)\right)\right]\\ =-\frac{1}{m}\overset{m}{\underset{i=1}{\sum }}\log\left(D\left(x^{\left(i\right)};\overset{⟶}{\partial_{D}}\right)\right)-\frac{1}{m}\overset{m}{\underset{i=1}{\sum }}\log\left(1-D\left(G\left({\overset{⟶}{z}}^{\left(i\right)};\overset{⟶}{\partial_{G}}\right);\overset{⟶}{\partial_{D}}\right)\right)\\ \approx -E_{x∼p_{\text{data}}}\log\left[D\left(x\right)\right]-E_{z∼p_{\text{prior}}}\log\left[1-D\left(G\left(z\right)\right)\right], \end{array} \end{array}$$

where *D*(*x*) is the Discriminator output (i.e., the probability of realism of the input *x*), *G*(*z*) is the output of the Generator network for random vector input *z* (i.e., an artificial image), pdata is the distribution followed by the data input (in these images it will be a very high dimensional distribution that can only be indirectly and approximately modeled by GAN), and pprior the prior distribution from which we sample to get the random vector at the Generator input. Since Discriminator predicts probability and therefore *D*(*x*) ∈ [0, 1], it follows that to minimize its cost function, Discriminator must learn to assign a high probability to samples labeled 1 (derived from the set of training data) and low on those generated by the Generator [21].

The Generator network, in turn, tries to “trick” the Discriminator so that the chances it assigns to the artificial samples at its output are high. It aims to maximize the second term of the Discriminator cost function - after all, only this term can affect the Discriminator's cost function to increase it. Therefore, the following will apply to the Generator [8]:

(3) $$\begin{array}{c} \begin{array}{c} J_{G}\left(\overset{⟶}{\partial_{G}},\overset{⟶}{\partial_{D}}\right)=\frac{1}{m}\overset{m}{\underset{i=1}{\sum }}\left[\left(1-y^{\left(i\right)}\right)\log\left(1-h\left(x^{\left(i\right)};\overset{⟶}{\partial }\right)\right)\right]\\ =\frac{1}{m}\overset{m}{\underset{i=1}{\sum }}\left[\log\left(1-D\left(G\left({\overset{⟶}{z}}^{\left(i\right)};\overset{⟶}{\partial_{G}}\right);\overset{⟶}{\partial_{D}}\right)\right)\right]\\ =\frac{1}{m}\overset{m}{\underset{i=1}{\sum }}\log\left(1-D\left(G\left({\overset{⟶}{z}}^{\left(i\right)};\overset{⟶}{\partial_{G}}\right);\overset{⟶}{\partial_{D}}\right)\right)\\ \approx E_{z∼p_{\text{prior}}}\log\left[1-D\left(G\left(z\right)\right)\right], \end{array} \end{array}$$

where the negative sign at the beginning has now been removed as the Generator tries by minimizing its cost function to increase that of the Discriminator, while all other sizes are as before. Because the first term of the equation depends only on the training data set, the above Generator cost function is declared as negative of the Discriminator cost function [22, 23]:

(4) $$\begin{array}{c} J_{G}\left(\overset{⟶}{\partial_{G}},\overset{⟶}{\partial_{C}}\right)=-J_{D}\left(\overset{⟶}{\partial_{C}},\overset{⟶}{\partial_{G}}\right). \end{array}$$

Focusing on the continuous 1-Lipschitz function *f*, in the proposed GAN is the Discriminator network itself, which, taking an image, *x*, is called upon to give a real number. Therefore, the function will be

(5) $$\begin{array}{c} c:X⟶\mathbb{R},{\left\|c\right\|}_{L}\leq 1. \end{array}$$

To successfully approach a neural network with trainable parameters ∼*θ* a continuous 1-Lipschitz function, the measure of some of the network output derivatives in terms of trainable parameters must be at most 1 at each point in the domain. Thus, the Discriminator neural network must satisfy the following continuity condition to be a 1-Lipschitz continuous function [24, 25]:

(6) $$\begin{array}{c} \nabla_{{\overset{⌢}{\partial }}_{C}}C{\left(x;\overset{⟶}{\partial_{C}}\right)}_{2}\leq 1\forall x\in X↔{\left\|c\right\|}_{L}\leq 1. \end{array}$$

This condition enforcement ensures that the cost function is valid when measuring the allocation distance. It is continuous and differentiable and does not increase too fast. The proposed model introduces a normalization term that imposes a penalty when the norm of some of the output derivatives of Discriminator concerning its input is greater than 1 so that [21]

(7) $$\begin{array}{c} {\text{reg}}_{GP}={\left(\nabla_{{\overset{⌢}{\partial }}_{C}}C{\left(\tilde{x};\tilde{x}\right)}_{2}-1\right)}^{2}, \end{array}$$

and so, the cost functions that the two neural networks try to minimize will be [8, 21, 22]:

(8) $$\begin{array}{c} \begin{array}{c} J_{C}\left(\overset{⟶}{\partial_{C}},\overset{⟶}{\partial_{G}}\right)=-\frac{1}{m}\overset{m}{\underset{i=1}{\sum }}\left[C\left(x^{\left(i\right)};\overset{⟶}{\partial_{C}}\right)\right]+\frac{1}{m}\overset{m}{\underset{i=1}{\sum }}\left[C\left(G\left({\overset{⟶}{z}}^{\left(i\right)};\overset{⟶}{\partial_{G}}\right);\overset{⟶}{\partial_{C}}\right)\right]+{\hat{\lambda }}_{GP}*reg_{GP}\\ =-\frac{1}{m}\overset{m}{\underset{i=1}{\sum }}\left[C\left(x^{\left(i\right)};\overset{⟶}{\partial_{C}}\right)\right]+\frac{1}{m}\overset{m}{\underset{i=1}{\sum }}\left[C\left(G\left({\overset{⟶}{z}}^{\left(i\right)};\overset{⟶}{\partial_{G}}\right);\overset{⟶}{\partial_{C}}\right)\right]\\ +\lambda_{GP}*\frac{1}{m}\overset{m}{\underset{i=1}{\sum }}\left[{\left(\nabla_{\overset{⟶}{\partial_{C}}}C{\left(\varepsilon *x+\left(1-\varepsilon \right)*\hat{x};\overset{⟶}{\partial_{C}}\right)}_{2}-1\right)}^{2}\right]\\ \approx -E_{x∼p_{\text{data}}}\left[C\left(x\right)\right]+E_{z∼p_{\text{priar}}}\left[C\left(G\left(z\right)\right)\right]+{\hat{\lambda }}_{GP}*E_{\tilde{x}∼p_{\tilde{x}}}\left[{\left(\nabla_{\tilde{x}}C{\left(\tilde{x}\right)}_{2}-1\right)}^{2}\right]. \end{array} \end{array}$$

To model the sequence of input symbols under a single framework, we propose in this work the use of optimal attention mechanisms both qualitatively and computationally. The proposed sparse attention mechanism requires much less memory, is faster, achieves better performance, and requires fewer training steps than intensive attention due to incorporating appropriate assumptions into its architectural design.

In particular, the quadratic complexity of attention is due to the calculation of the table [17, 23]:

(9) $$\begin{array}{c} M_{Q,K}=Q\cdot K^{T},\;\in {\mathbb{R}}^{N_{X}\times N_{Y}}. \end{array}$$

Instead, we propose multidimensional attention mechanisms in this work. In each Step i, attention is limited to a set of predefined positions given by a mask:

(10) $$\begin{array}{c} A_{i}\in {\left\{0,1\right\}}^{N_{X}\times N_{Y}}. \end{array}$$

In each Step i, we calculate

(11) $$\begin{array}{c} M_{Q,K}^{i}\left[a,b\right]=\left\{\begin{array}{c} M_{Q,K}\left[a,b\right],A^{i}\left[a,b\right]=1,\\ -\infty ,A^{i}\left[a,b\right]=0. \end{array}\right. \end{array}$$

In addition, using information flow charts and the two-dimensional geometry conservation mechanism, we construct a sparse multistep attention layer that can model any dependencies on the input data and respects the native pixel locality in a video. An indicative representation of spherical 2-D points far away from the sphere is very unlikely to fall in the same area at all random rotations, which is reversed for very close points to the sphere, as shown in Figure 2.

This process is directly related to the tendency of the softmax function to yield sparse distributions. So, by this logic, we argue that the dense models produce sparse attention maps:

(12) $$\begin{array}{c} E\left(X_{k:n}\right)\leq \mu +\sigma \sqrt{\frac{k-1}{n-k+1}}. \end{array}$$

Based on the above relation, we can prove the rarity of the probabilistic distributions obtained from softmax [21–23]:

(13) $$\begin{array}{c} \frac{e^{E\left(X_{k:n}\right)}}{\sum_{i=1}^{n}e^{E\left(X_{i}\right)}}\leq \frac{e^{\mu +\sigma \sqrt{k-1/n-k+1}}}{\sum_{i=1}^{n}e^{E\left(X_{i}\right)}}=\frac{e^{\mu +\sigma \sqrt{k-1/n-k+1}}}{ne^{\mu }}. \end{array}$$

which with limits *μ* = 0 and *σ*2 = 1 can be calculated as

(14) $$\begin{array}{c} \begin{array}{c} E\left(\frac{e^{X_{k:n}}}{\sum_{i=1}^{n}e^{X_{i:n}}}\right)\leq \epsilon ,\\ \frac{e^{\sqrt{k-1/n-k+1}}}{n}\leq \epsilon \overset{n\in \geq 1}{⇌}\sqrt{\frac{k-1}{n-k+1}}\leq ln\left(n\epsilon \right)\\ k\leq \frac{1+\left(n+1\right){\text{ln}}^{2}\left(n\epsilon \right)}{1+{\text{ln}}^{2}\left(n\epsilon \right)}. \end{array} \end{array}$$

The challenge in multistep attention mechanisms is the design of dual masks for each step. This paper uses an information theory tool to successfully design sparse attention patterns. Specifically, information flow graphs are used, which are guided, acyclic graphs that model the flow of network information into graphs of distributed systems. For our problem, these graphs show the flow of information between the attention steps and the corresponding transformations that follow. The most common of the proposed transformations are [8, 22, 23]:

(15) $$\begin{array}{c} \left\{\begin{array}{c} F\left(q_{i}\right)=\left[q_{i};\frac{1}{2},\ldots ;\frac{1}{2}\right],G\left(k_{i}\right)=\left[Uk_{i};Uk_{i2}^{2};\ldots ;Uk_{i2}^{2}\right],\\ F\left(q_{i}\right)=\left[q_{i};0\right],G\left(k_{i}\right)=\left[k_{i};\sqrt{M_{K}^{2}-k_{i2}^{2}}\right],\\ F\left(q\right)=\frac{M_{K}}{{\left\|q\right\|}_{2}}\cdot \left[q;0\right],G\left(k\right)=\left[k;\sqrt{M_{K}^{2}-{\left\|k\right\|}_{2}^{2}}\right]. \end{array}\right. \end{array}$$

To smooth out the deformations resulting from the above transformations, the proposed system allows the focus on the previous and next stage, as shown in Figure 3 below:

For each set of masks {*A*^1^,…, *A*^*p*^} we make a polymer graph *G*(*V*={*V*^0^, *V*^1^,…, *V*^*p*^}, *E*) where the edges between *V*^*i*^, *V*^*i*+1^ are determined by the mask Mi. Thus, a sparse pattern has complete information if the relevant information graph has a path from each node a ∈ V0 to each node *b*∈ Vp. So, in addition to the computational improvement of the dense attention mechanism, the sparse attention mechanisms also achieve better results due to the integration of prior knowledge of locality into the information flow chart.

Our mechanism has O($n\sqrt{n}$) memory complexity and speed, significantly reducing the square complexity of intensive attention. The probability distributions created within the attention map make a new method for reversing the proposed attention GAN. Essentially, the proposed technique provides the methodology for evaluating the boundaries of indeterminate forms so that by applying them, an indefinite form can be quickly assessed by substitution [21, 22]:

(16) $$\begin{array}{c} \underset{h⟶0^{+}}{\lim}\frac{1}{h}\int_{x_{j}}^{x_{j}+h}f\left(x|\theta \right)\text{d}x=\underset{h⟶0^{+}}{\lim}\frac{d/\text{d}h\int_{x_{j}}^{x_{j}+h}f\left(x|\theta \right)\text{d}x}{\text{d}h/\text{d}h}\\ =\underset{h⟶0^{+}}{\lim}\frac{f\left(x_{j}+h|\theta \right)}{1}\\ =f\left(x_{j}|\theta \right). \end{array}$$

Then,

(17) $$\begin{array}{c} {\text{argmax}}_{\theta }ℒ\left(\theta |x_{j}\right)={\text{argmax}}_{\theta }\left[\underset{h⟶0^{+}}{\text{lim}}ℒ\left(\theta |x\in \left[x_{j},x_{j}+h\right]\right)\right]\\ ={\text{argmax}}_{\theta }\left[\underset{h⟶0^{+}}{\text{lim}}\frac{1}{h}\int_{x_{j}}^{x_{j}+h}f\left(x|\theta \right)\text{d}x\right]\\ ={\text{argmax}}_{\theta }f\left(x_{j}|\theta \right). \end{array}$$

Therefore,

(18) $$\begin{array}{c} {\text{argmax}}_{\theta }ℒ\left(\theta |x_{j}\right)={\text{argmax}}_{\theta }f\left(x_{j}|\theta \right), \end{array}$$

and so, maximizing the probability density in *x*_*j*_ equals maximizing the probability of that observation in *x*_*j*_, thus creating the method of the proposed attention.

As a novel approach, this technique is an intelligent advanced mechanism that uses attention mechanisms but does not have a square complexity of memory and time in terms of the input size. So, it is possible to accurately detect obscene and primarily sexual content in streaming online video conferencing software.

## 4. Scenarios and Results

The research was also conducted to assess the likelihood that the user will engage in abnormal behavior related to displaying inappropriate content [7, 26]. A specialized scenario was implemented to model the proposed system to calibrate the user's actions during the live video stream about an activity that might be considered provocative or inappropriate. This process was based on the technique of visual flow, which involves the movement of objects between successive snapshots of a video, which arises due to the action of objects. Sparse optical flow detects characteristic points, such as angles and edges of the image, and their monitoring in successive snapshots, while dense visual flow refers to the estimation of the motion vectors of the whole image, i.e., all pixels.

More specifically, the scenario assumes that the optical flux is a standard estimate where the position of each point is defined using a square polynomial of the form *f*_1_(*x*)=*x*^*T*^*A*_1_*x*+*b*^*T*^*x*+*c*_1_, where Α is a symmetric array, *b* vector, and *c* graded number. An adjustment of least squares determines the coefficients. Respectively for the second scene, it applies that [27–29]:

(19) $$\begin{array}{c} f_{2}\left(\text{x}\right)=f_{1}\left(\text{x}-\text{d}\right). \end{array}$$

Therefore, we have

(20) $$\begin{array}{c} \begin{array}{c} \begin{array}{c} f_{2}\left(x\right)=f_{1}\left(x-d\right)\\ ={\left(x-d\right)}^{T}{\text{A}}_{1}\left(x-d\right)+{\text{b}}_{1}^{T}\left(x-d\right)+c_{1} \end{array}\\ ={\text{x}}^{T}{\text{A}}_{1}x+{\left({\text{b}}_{1}-2{\text{A}}_{1}\text{d}\right)}^{T}x+{\text{d}}^{T}{\text{A}}_{1}d-{\text{b}}_{1}^{T}d+c_{1}\\ ={\text{x}}^{T}{\text{A}}_{2}x+{\text{b}}_{2}^{T}x+c_{2}. \end{array} \end{array}$$

If the coefficients of the square polynomials are equated, we have

(21) $$\begin{array}{c} \begin{array}{c} {\text{A}}_{2}{\text{A}}_{1},\\ {\text{b}}_{2}={\text{b}}_{1}-2{\text{A}}_{1}d,\\ c_{2}={\text{d}}^{T}{\text{A}}_{1}d-{\text{b}}_{1}^{T}d+c_{1}. \end{array} \end{array}$$

And since A is reversible, we have

(22) $$\begin{array}{c} \text{d}=-\frac{1}{2}{\text{A}}_{1}^{-1}\left({\text{b}}_{2}-{\text{b}}_{1}\right). \end{array}$$

This condition does not apply to the entire image signal, as there is no universal permutation. Thus, the universal polynomial equation is converted to local with coefficients *A*1(*x*), *b*1(*x*), and *c*1(*x*). Even the condition *A*1 = A2 is practically not valid, so it is estimated as [27, 28]

(23) $$\begin{array}{c} \text{A}\left(\text{x}\right)=\frac{{\text{A}}_{1}\left(\text{x}\right)+{\text{A}}_{2}\left(\text{x}\right)}{2}. \end{array}$$

Finally, we define

(24) $$\begin{array}{c} \Delta \text{bb}\left(\text{x}\right)=-\frac{1}{2}\left({\text{b}}_{2}\left(\text{x}\right)-{\text{b}}_{1}\left(\text{x}\right)\right). \end{array}$$

We have

(25) $$\begin{array}{c} \text{A}\left(\text{x}\right)\text{d}\left(\text{x}\right)=\Delta \text{b}\left(\text{x}\right), \end{array}$$

where *d*(*x*) now has local power and is not universal. Finally, to improve the accuracy, we can apply this condition to the whole neighboring area and not to each pixel separately, minimizing the relationship [13, 23, 26]:

(26) $$\begin{array}{c} \underset{\Delta \text{x}\in I}{\sum }w\left(\Delta x\right){\left\|\text{A}\left(\text{x}+\Delta \text{x}\right)\text{d}\left(\text{x}\right)-\Delta \text{b}\left(\text{x}+\Delta \text{x}\right)\right\|}^{2}, \end{array}$$

where w(∆*x*), weight function of adjacent points. So, the field of view is ultimately

(27) $$\begin{array}{c} \text{d}\left(\text{x}\right)={\left(\sum w{\text{A}}^{T}A\right)}^{-1}\sum w{\text{A}}^{T}\text{b}\text{.} \end{array}$$

So, the algorithm's operation is based on the minimization of a function that includes an information term using the L1 norm and a normalization term using the optical fluctuation. Brightness constancy assumption is initially considered as

(28) $$\begin{array}{c} \frac{d}{dt}I\left(x\left(t\right),y\left(t\right),t\right)=0, \end{array}$$

where *I*(*x*(*t*), *y*(*t*), *t*) the video and (*x*(*t*), *y*(*t*)) the trajectory of a point in the image. Applying the chain rule results in

(29) $$\begin{array}{c} \nabla I\cdot \left(\dot{x},\dot{y}\right)+\frac{\partial }{\partial t}I=0. \end{array}$$

It is also defined as the speed of the orbits:

(30) $$\begin{array}{c} \text{u}\left(x,y\right)=\left(u_{1}\left(x,y\right),u_{2}\left(x,y\right)\right), \end{array}$$

and the visual flow is committed to locating the reference point, which in the resulting case is the inappropriate material:

(31) $$\begin{array}{c} \nabla I\cdot u+\frac{\partial }{\partial t}I=0. \end{array}$$

For each point in the image, this equation has 2 unknown variables, the velocity components *u*. Therefore, the system does not have a unique solution. To solve this problem, we use a smoothing term to force the normalization of *u*.

In the proposed model, the solution is performed by minimizing the energy function resulting from the sum of the variability of *u* and the term L1 when the following function is applied [13, 17, 21]:

(32) $$\begin{array}{c} E\left(\text{u}\right)=\int_{\Omega }\left|\nabla u_{1}\right|+\left|\nabla u_{2}\right|+\lambda \left|\rho \left(\text{u}\right)\right|. \end{array}$$

The minimization process for finding *u* is performed for different image scales. The vector *u* is initially calculated for large scales, initial values for the more minor scales. Thus, the vector *u* is gradually determined more accurately.

Finally, for the proposed algorithm to better render the classification coded features, the Gaussian Mixture Model (GMM) is first calculated to model the distributions of video descriptions. The vectors then encode the slope of the logarithmic probability of the features according to the GMM parameters. Let Χ = {*x*1, *x*2, *x*t} the n-dimensional features. The GMM parameters are estimated based on these characteristics: weights, averages, and variability. Accordingly, the logarithmic probability slopes for the GMM parameters are calculated as follows [11, 30, 31]:

(33) $$\begin{array}{c} \nabla_{\alpha_{k}}\log\;p\left(X\right)=\overset{t}{\underset{i=1}{\sum }}\nabla_{\alpha_{k}}\log\;p\left(x_{t}\right),\\ \nabla_{\mu_{k}}\log\;p\left(X\right)=\overset{t}{\underset{i=1}{\sum }}\nabla_{\mu_{k}}\log\;p\left(x_{t}\right),\\ \nabla_{\sigma_{k}}\log\;p\left(X\right)=\overset{t}{\underset{i=1}{\sum }}\nabla_{\sigma_{k}}\log\;p\left(x_{t}\right), \end{array}$$

where from the sum of the three vectors results [31, 32]:

(34) $$\begin{array}{c} FV=\left[\nabla_{\alpha_{k}}\text{log}p\left(X\right),\nabla_{\mu_{k}}\text{log}p\left(X\right),\nabla_{\sigma_{k}}\text{log}p\left(X\right)\right]. \end{array}$$

The pornography database [4, 6, 19, 30], which contains nearly 80 hours of 400 pornographic and 400 non-pornographic videos, was used to locate the scenes of inappropriate material. The pornographic material comes from relevant sites that host only such material. At the same time, it should be emphasized that the set consists of various types of pornography and depicts actors of many ethnicities. Respectively, the non-pornographic content came from browsing the web with general-purpose videos.

During pre-processing, all videos were initially segmented into shots. A basic (non-inappropriate) frame was used to summarize the content of the picture into a still image. Some typical static images from photos contained in this dataset are shown in Figure 4 below [1, 5, 30].

All the exterior shots, such as beach shots, were removed, and only indoor pictures were used. In total, 12,182 videos were used, of which 6,743 were inappropriate, and 5,439 were inappropriate.

The video observations based on the density estimation were given in time-series images, where the *x*-axis symbolizes time. In probability and statistics, density estimation is constructing an estimate of an unobservable underlying probability density function using observed data. The unobservable density function describes the distribution of a vast population; the data are typically viewed as a random sampling from that population. Density estimation techniques such as Parzen windows and various data clustering techniques, including vector quantization, are used. The simplest method for estimating density is to use a rescaled histogram. In this paper, for uniformity and comparison of the results, along with the pictures of the model estimation, a heuristic method was used based on the images of the experts' observations and their votes in terms of content for each scene. Models trained with batch learning in the material in question were used as specialists. This procedure was done for each video, based on the total time in seconds that each category lasted within the video [6, 30].

The 10-fold cross-validation method was used for the experimental evaluation. In contrast, the Mean Average Precision (MAP) and Accuracy Rate (AcR) were used as the scoring measure, where most evaluators take the final class of the examined video. Finally, the ROC Curve and F-measure metrics displayed the results. The results of the procedure are shown in Table 1 below.

As can be seen from the table above, the results look pretty satisfactory. In some cases, the model finds it challenging to locate the noPorn category, slightly reducing its overall performance. This is because the vector representations are identical. Although experimentally, this did not reduce the performance for the problems tested, there may be other problems with a drop. Even more importantly, this limits its use to situations where the number of classes is multiple.

For this problem, a simple solution was used to replace the imaging function to group vectors with short Euclidean distances or large internal products to have data located in some lower norm sphere or even data without geometric constraints. The results of the procedure are shown in Table 2 below.

As can be seen, alternative display schemes achieve much better results without imposing such strong constraints on the nature of the input data. The main problem of the proposed solution is that it requires network retraining and, therefore, cannot operate on pretrained networks. This significantly reduces its usefulness as retraining costs are vast, and the chances of mastering sparse attention mechanisms are slim.

The groups are created randomly in random attention, and the attention occurs within the group. To increase the probability of success of the method, we repeat the process a few times. For this reason, we propose a comparison model, the randomization, which can be used to create sparse models that do not require retraining. As shown in Table 3 below, the model in question achieves impressive results.

It seems that this model can begin the search to find attention mechanisms that do not require retraining.

## 5. Conclusions

In this work, we proposed and studied solutions for efficient attention mechanisms. The methods presented are based on either predetermined sparse patterns or dynamic dilution. The advanced technique first introduced in the literature suggests a GAN assisted by attention mechanisms, which can speed up and even be more efficient, allowing for faster processing and fewer memory requirements. The methodology is used in a case study to deal with incidents of fair or unfair exposure to offshore content to underage students during distance learning in online education video conference applications. A significant disadvantage of the proposed method is that it requires an extensive bandwidth network.

Changes that can lead to simpler variants of attention that operate without imposing restrictions on attention inputs are critical future developments in this work. Also, the search for even more efficient computing methods and, in general, the solutions that can significantly improve the performance of solving complex real-time problems like the one studied. Finally, it is crucial to investigate how an external classification scheme can be implemented that can achieve high acceleration for a sufficiently large input size.

## Figures and Tables

**Figure 1:** The binary Cross-Entropy loss function for real (left) and fake (right) data.

**Figure 2:** Spherical 2-D case study.

**Figure 3:** Depiction of transformer attention.

**Figure 4:** Pornography database.

**Table 1:** Performance metrics of the classification process - 1.

	MAP	AcR	ROC curve	F-measure
Porn	92.532	91.912	95.004	92.301
noPorn	88.024	89.031	88.558	89.065

**Table 2:** Performance metrics of the classification process - 2.

	MAP	AcR	ROC curve	F-measure
Porn	95.871	95.568	95.997	96.163
noPorn	92.958	91.597	91.869	91.733

**Table 3:** Performance metrics of the classification process - 3.

	MAP	AcR	ROC curve	F-measure
Porn	99.220	99.118	99.672	99.258
noPorn	98.487	98.596	98.604	98.599

## Data Availability

The data are available at https://sites.google.com/site/pornographydatabase/

## References

[1] Gangwar A., Fidalgo E., Alegre E., González-Castro V. Pornography and child sexual abuse detection in image and video: a comparative evaluation.

[2] Moustafa M. (2015). Applying Deep Learning to Classify Pornographic Images and Videos. https://arxiv.org/abs/1511.08899.

[3] Perez M., Avila S., Moreira D. (2017). Video pornography detection through deep learning techniques and motion information. *Neurocomputing*.

[4] Wehrmann J., Simões G. S., Barros R. C., Cavalcante V. F. (2018). Adult content detection in videos with convolutional and recurrent neural networks. *Neurocomputing*.

[5] Vitorino P., Avila S., Perez M., Rocha A. (2018). Leveraging deep neural networks to fight child pornography in the age of social media. *Journal of Visual Communication and Image Representation*.

[6] Ou X., Ling H., Yu H., Li P., Zou F., Liu S. (2017). Adult image and video recognition by a deep multicontext network and fine-to-coarse strategy. *ACM Transactions on Intelligent Systems and Technology*.

[7] Yuan K., Tang D., Liao X. Stealthy porn: understanding real-world adversarial images for illicit online promotion. *2019 IEEE Symposium on Security and Privacy (SP)*.

[8] Li D., Wang R., Chen P., Xie C., Zhou Q., Jia X. (2021). Visual feature learning on video object and human action detection: a systematic review. *Micromachines*.

[9] Xing L., Demertzis K., Yang J. (2020). Identifying data streams anomalies by evolving spiking restricted Boltzmann machines. *Neural Computing & Applications*.

[10] Jing L., Tian Y. (2021). Self-supervised visual feature learning with deep neural networks: a survey. *IEEE Transactions on Pattern Analysis and Machine Intelligence*.

[11] Ali S. T., Goyal K., Singhai J. Moving object detection using self adaptive Gaussian Mixture Model for real time applications.

[12] Kasthuri Arachchi S. P., Shih T. K., Hakim N. L. (2020). Modelling a spatial-motion deep learning framework to classify dynamic patterns of videos. *Applied Sciences*.

[13] Vishwanath B., Rose K. Spherical video coding with geometry and region adaptive transform domain temporal prediction.

[14] Duboyskii I., Shabanova A., Sivchenko O., Usina E. (2020). Architecture of cross-platform videoconferencing system with automatic recognition of user emotions. *IOP Conference Series: Materials Science and Engineering*.

[15] Vondrick C., Pirsiavash H., Torralba A. (2016). Generating videos with scene dynamics. *Advances in Neural Information Processing Systems*.

[16] Tulyakov S., Liu M.-Y., Yang X., Kautz J. (2017). MoCoGAN: Decomposing Motion and Content for Video Generation. https://arxiv.org/abs/1707.04993.

[17] Murphy K. P. (2012). *Machine Learning: A Probabilistic Perspective*.

[18] Feng J., Feng X., Chen J. (2020). Generative adversarial networks based on collaborative learning and attention mechanism for hyperspectral image classification. *Remote Sensing*.

[19] Moreira D., Avila S., Perez M. (2016). Pornography classification: the hidden clues in video space-time. *Forensic Science International*.

[20] Corley I., Lwowski J., Hoffman J. (2020). DomainGAN: Generating Adversarial Examples to Attack Domain Generation Algorithm Classifiers. http://arxiv.org/abs/1911.06285.

[21] Gui J., Sun Z., Wen Y., Tao D., Ye J. (2020). A Review on Generative Adversarial Networks: Algorithms, Theory, and Applications. http://arxiv.org/abs/2001.06937.

[22] Dash A., Ye J., Wang G. (2021). A review of generative adversarial networks (GANs) and its applications in a wide variety of disciplines -- from medical to remote sensing. http://arxiv.org/abs/2110.01442.

[23] S. K., Durgadevi M. Generative Adversarial Network (GAN): a general review on different variants of GAN and applications. *2021 6th International Conference on Communication and Electronics Systems (ICCES)*.

[24] Hu G.-D. (2006). Observers for one-sided Lipschitz non-linear systems. *IMA Journal of Mathematical Control and Information*.

[25] Loeb I. (2013). Lipschitz functions in constructive reverse mathematics. *Logic Journal of IGPL*.

[26] Caetano C., Avila S., Schwartz W. R., Guimarães S. J. F., Araújo A. d. A. (2016). A mid-level video representation based on binary descriptors: a case study for pornography detection. *Neurocomputing*.

[27] Cai Z., Huang H., Wu W., Ma X., Hu X. Detecting gathering incident of video surveillance based on plane geometry.

[28] He Y., Ye Y., Hanhart P., Xiu X. Motion compensated prediction with geometry padding for 360 video coding.

[29] Oh H., Lee S. (2016). Visual presence: viewing geometry visual information of UHD S3D entertainment. *IEEE Transactions on Image Processing*.

[30] Avila S., Thome N., Cord M., Valle E., Araújo A. (2013). Pooling in image representation: the visual codeword point of view. *Computer Vision and Image Understanding*.

[31] Satriyanto N., Munir R. Dynamic background video forgery detection using Gaussian mixture model.

[32] He W., Yu R., Zheng Y., Jiang T. Image denoising using asymmetric Gaussian mixture models.

